The article "Predictive Value of MPV and Plasma NT-ProBNP Combined with the Simplified Geneva Scale for the Prognosis of Acute Pulmonary Embolism" was retracted in 2023. Reasons: signs of a paper mill; suspected computer-generated content; unreliable results or conclusions; lack of ethics approval or compliance.

# Predictive Value of MPV and Plasma NT-ProBNP Combined with the Simplified Geneva Scale for the Prognosis of Acute Pulmonary Embolism

**DOI:** 10.1155/2021/1292921

**Published:** 2021-10-19

**Authors:** Jing Wang, Lu Wang, Ling Jin, Xiaolei Rong, Xueshuang Tang, Haina Guo, Xiaochuan Liu, Lei Shi, Guilu Tao

**Affiliations:** ^1^Department of Wound Repairment and Intervention, The Second Affiliated Hospital of Dalian Medical University, Dalian, Liaoning 116000, China; ^2^Department of Internal Medicine, The Second Affiliated Hospital of Dalian Medical University, Dalian, Liaoning 116000, China; ^3^Department of General Surgery, The Second Affiliated Hospital of Dalian Medical University, Dalian, Liaoning 116000, China

## Abstract

**Objective:**

To explore the predictive value of mean platelet volume (MPV) and plasma *N*-terminal probrain natriuretic peptide (NT-ProBNP) combined with a simplified Geneva scale for the prognosis of acute pulmonary embolism (APE).

**Methods:**

The clinical data of 68 patients with APE admitted to our hospital from October 2017 to October 2019 were collected. According to the prognosis, the patients were divided into a good prognosis group (*n* = 45) and a poor prognosis group (*n* = 23). The clinical data, laboratory clinical indexes, and simplified Geneva scale scores were recorded for the two groups. The risk factors of poor prognosis were analyzed by binary multivariate logistic regression analysis; the predictive ability of each index on the prognosis of patients with APE was analyzed by the ROC curve.

**Results:**

The incidences of deep vein thrombosis, diabetes, and hyperlipidemia in the poor prognosis group were higher than those in the good prognosis group (*P* < 0.05). PLT, platelet distribution width (PDW), MPV, and plasma NT-ProBNP in the poor prognosis group were higher than those in the good prognosis group (*P* < 0.05). The simplified Geneva scale score of the poor prognosis group was higher than that of the good prognosis group (*P* < 0.05). PDW, MPV, plasma NT-ProBNP, and simplified Geneva scale were all independent risk factors for the poor prognosis of APE patients (*P* < 0.05). The AUC of MPV in predicting the prognosis of APE patients was 0.818 (95% CI: 0.712–0.925). When the optimal cutoff value was 0.571, the sensitivity was 77.1%, and the specificity was 80.0%. The AUC of plasma NT-ProBNP in predicting the prognosis of APE patients was 0.762 (95% CI: 0.634–0.891). When the optimal cutoff value was 0.475, the sensitivity was 71.5%, and the specificity was 76.0%. The AUC of the simplified Geneva scale in predicting the prognosis of APE patients was 0.749 (95% CI: 0.618–0.879). When the optimal cutoff value was 0.469, the sensitivity was 82.9%, and the specificity was 64.0%. The AUC of MPV and plasma NT-ProBNP combined with the simplified Geneva scale in predicting the prognosis of APE patients was 0.907 (95% CI: 0.826–0.988). When the optimal cutoff value was 0.726, the sensitivity was 88.6%, and the specificity was 84.0%.

**Conclusion:**

MPV, plasma NT-ProBNP, and simplified Geneva scale have a certain predictive value for the prognosis of APE. Compared with a single index, the combination of the three indexes has a significant improvement in predicting the prognosis of APE and has better clinical value.

## 1. Introduction

Acute pulmonary embolism (APE) refers to a variety of emboli that block the pulmonary artery and its branches, leading to pulmonary circulation disorders, resulting in a variety of pathological and physiological changes. APE is mainly manifested as sudden chest pain, dyspnea, hemoptysis, and other manifestations. It has a rapid onset and rapid development and has the characteristics of low specificity and poor prognosis [1, 2]. In recent years, the number of patients suffering from APE has been increasing. According to the survey, the incidence rate of APE in organic heart disease is about 5%–10%; the incidence rate of APE in the total number of hospitalizations is about 2.5%–6.5%; and the incidence rate can be as high as 10%–14% in the areas with high incidence [3]. In my country, APE has become the third-largest cardiovascular disease in clinical practice, second only to coronary heart disease and hypertension, which seriously endangers the quality of life and health of patients [4]. Therefore, it is of great significance to evaluate the prognosis of APE patients as soon as possible and adopt scientific and reasonable countermeasures to deal with the disease.

Mean platelet volume (MPV) is an indicator of platelet function, which can reflect the production and activation of platelets, and plays an important role in the diagnosis of acute pancreatitis, colorectal cancer, respiratory diseases, and other diseases [5–7]. *N*-terminal pro-brain natriuretic peptide (NT-ProBNP) is a metabolic substance in the process of myocardial cells producing BNP, which can reflect the state of the body's heart function. The higher the level of NT-ProBNP, the larger the area of the embolized blood vessel, the more severe the degree of right heart dysfunction and myocardial damage, the worse the prognosis of patients. NT-ProBNP has a slower clearance in the blood and a long half-life, and the concentration of NT-ProBNP in plasma is higher than that of BNP, and it has no biological activity. Its detection is not easy to be affected by drugs, and the determination results are more accurate and sensitive and have been applied in the diagnosis and prognosis of a variety of diseases [8]. Studies have shown that when the level of NT-probNP is normal, the possibility of acute pulmonary embolism as the cause of death in hospitalized patients can be basically excluded, with specificity reaching 97%–100% [9]. The simplified Geneva scale is a clinical possibility evaluation tool for PE developed by Klok after being simplified based on symptoms and risk factors. Most of the simplified Geneva scale are objective indicators, and risk factors such as advanced age, fracture, and heart rate are added. The quantified scores are based on the corresponding scores. The sensitivity, diagnostic accuracy, and consistency of these scales are better than that of the Wells scale, which has been widely used in clinical practice. The simplified Geneva scale is easy to operate, objective, and efficient; it may be more suitable for emergency patients and can be popularized and used in primary hospitals [10].

The objective of this study was to investigate the predictive value of MPV and plasma NT-ProBNP combined with a simplified Geneva scale in predicting the prognosis of APE.

## 2. Materials and Methods

### 2.1. Research Object

The clinical data of 68 patients with APE admitted to our hospital from October 2017 to October 2019 were collected. Among them, 39 were males, and 29 were females, with an average age of (56.23 ± 11.86) years.

#### 2.1.1. Diagnostic Criteria

① Symptoms: the clinical manifestations were complex and diverse, with low specificity, most of which were dyspnea, chest pain, syncope, hemoptysis, and other symptoms. ② Signs: mainly the signs of the respiratory system and circulatory system, manifested as increased respiratory rate (>20 beats/min), increased heart rate (>90 beats/min), cyanosis, and hypotension. ③ Pulmonary artery CTA: the image conforms to the following manifestations: direct signs: (1) partial thromboembolism, the thrombus was free in the vascular lumen, and the surrounding contrast agent surrounds and presents a circular low-density shadow. (2) Complete thromboembolism, the distal blood vessels were not visible, and the official cavity was completely blocked into a cup or irregular club. (3) Annular mural thrombus, showing mural filling defect [11].

#### 2.1.2. Inclusion Criteria

The diagnostic criteria of APE were met. All patients were diagnosed by CT angiography, radionuclide pulmonary ventilation/perfusion scan, and pulmonary artery angiography. Onset time <24 h; age ≥18 years; and the medical history data were complete.

#### 2.1.3. Exclusion Criteria

The exclusion criteria were as follows: chronic thromboembolic pulmonary hypertension; anticoagulant or thrombolytic therapy had been performed before admission; heart, liver, and kidney insufficiency; severe respiratory infections; severe blood system disease; blood indicators that have not met the requirements; previous cerebral infarction; patients who had undergone coronary artery bypass grafting or stenting; pregnant and lactating women; mentally ill; and unable to follow visitors.

#### 2.1.4. Ethics

In this study, clinical data of study subjects were retrospectively analyzed, and since there were no intervention activities for patients in this study, the process of signing informed consent could be exempted in this study.

### 2.2. Research Methods

All patients were followed up for 1 month, and the prognosis of the patients after discharge from the hospital was recorded. Poor prognosis was defined as adverse events such as death (death due to various reasons), deterioration of the disease (increased severity of the disease), APE recurrence (after recovery and discharge and readmission to APE), mechanical ventilation, and tracheal intubation. According to the prognosis, the patients were divided into a good prognosis group (*n* = 45) and a poor prognosis group (*n* = 23).

The clinical data of all patients were obtained from the hospital electronic medical record system, and the age, gender, body mass index (BMI), smoking history, drinking history, predisposing factors, and primary diseases of all patients were recorded.

The laboratory clinical indexes of the patients were recorded 24 h after admission: white blood cell count (WBC), red blood cell count (RBC), hemoglobin (Hb), platelet count (PLT), platelet distribution width (PDW), MPV, plasma NT-ProBNP, and so on.

The simplified Geneva scale score was recorded for all patients, with a total of 9 indicators, a total score of 0–10 points. The higher the score, the greater the risk of APE. The specific scoring operation of this scale was carried out by nurses in our department (see Table 1 for details).

### 2.3. Statistical Methods

SPSS 22.0 software was used for analysis. The measurement data that obey the normal distribution were expressed as mean ± standard deviation; *t*-test was used to analyze the comparison. Count data were expressed as a ratio, and *χ*^2^-test was used to analyze the comparison. The risk factors of poor prognosis were analyzed by binary multivariate logistic regression analysis; the predictive ability of each index on the prognosis of patients with APE was analyzed by ROC curve. *P* < 0.05 was statistically significant.

## 3. Results

### 3.1. Comparison of Clinical Data between the Two Groups

There was no significant difference between the two groups in age, gender, BMI, smoking history, drinking history, surgery or trauma, tumor, idiopathic factors, and other primary diseases such as hypertension, coronary heart disease, and chronic kidney disease (*P* > 0.05). The incidences of deep vein thrombosis, diabetes, and hyperlipidemia in the poor prognosis group were higher than those in the good prognosis group (*P* < 0.05; Table 2).

### 3.2. Comparison of Clinical Indexes between the Two Groups

There was no significant difference in WBC, RBC, and Hb between the two groups (*P* > 0.05). PLT, PDW, MPV, and plasma NT-ProBNP in the poor prognosis group were higher than those in the good prognosis group (*P* < 0.05; Figure 1).

### 3.3. Comparison of Clinical Scores between the Two Groups

The simplified Geneva scale score of the poor prognosis group was higher than that of the good prognosis group (*P* < 0.05; Figure 2).

### 3.4. Multivariate Analysis of Prognostic Factors in Patients with APE

Multivariate regression analysis showed that PDW, MPV, plasma NT-ProBNP, and simplified Geneva scale were all independent risk factors for poor prognosis of APE patients (*P* < 0.05; Table 3).

### 3.5. Prognostic Value of Each Index in Patients with APE

MPV, plasma NT-ProBNP, and simplified Geneva scale had high predictive value for the prognosis of APE patients. The AUC of MPV in predicting the prognosis of APE patients was 0.818 (95% CI 0.712–0.925). When the optimal cutoff value was 0.571, the sensitivity was 77.1%, and the specificity was 80.0%; The AUC of plasma NT-ProBNP in predicting the prognosis of APE patients was 0.762 (95% CI 0.634–0.891). When the optimal cutoff value was 0.475, the sensitivity was 71.5%, and the specificity was 76.0%. The AUC of the simplified Geneva scale in predicting the prognosis of APE patients was 0.749 (95% CI 0.618–0.879). When the optimal cutoff value was 0.469, the sensitivity was 82.9%, and the specificity was 64.0%; The AUC of MPV, and plasma NT-ProBNP combined with simplified Geneva scale in predicting the prognosis of APE patients was 0.907 (95% CI 0.826–0.988). When the optimal cutoff value was 0.726, the sensitivity was 88.6%, and the specificity was 84.0% (Table 4; Figure 3).

## 4. Discussion

As an acute and severe disease with frequent clinical occurrence, APE is characterized by atypical clinical manifestations, the rapid development of the disease, and poor prognosis; its prevalence of APE increases with age; and it has a higher risk of death [12]. The study by Konstantinides et al. [3] reported that the mortality rate of APE patients without treatment was about 30%, and the mortality rate of hospitalized APE patients was about 23.8%. We believe that the prognosis of APE patients is quite different. Even if the patients are treated actively, only some of them have a good prognosis, but some patients still have relapses or even die suddenly, which causes serious harm to the life and health of the patients. At this stage, the gold standard for clinical diagnosis of APE is pulmonary artery CTA. This method injects contrast medium into the pulmonary artery and judges APE based on whether the contrast medium filled in the pulmonary artery is complete, whether the blood flow is blocked, or uses the velocity of contrast agent in the pulmonary artery to determine APE. However, pulmonary artery CTA is traumatic, and its inspection cost is relatively high. So it is difficult to carry out this inspection method in primary hospitals. Therefore, it is of great significance to actively seek effective clinical indicators to evaluate the prognosis of APE patients.

The results of this study showed that the incidence of deep vein thrombosis, diabetes, and hyperlipidemia in the poor prognosis group were higher than those in the good prognosis group. This suggested that deep vein thrombosis, diabetes, and hyperlipidemia can all affect the prognosis of APE patients. The possible reasons are: when deep vein thrombosis is formed, the thrombus can fall off and can travel along the bloodstream to the lung, causing the blood vessel to block, which in turn leads to an increased risk of APE recurrence and poor prognosis. In addition, the blood of patients with diabetes and hyperlipidemia is often in a state of hypercoagulation; the blood of patients is relatively viscous, prone to the formation of thrombosis, and can damage the blood vessel wall, leading to the thrombus falling off, thereby affecting the prognosis of APE patients [13].

As a parameter indicating the volume and size of platelets, MPV can reflect the function of platelets and is closely related to the production of thrombus. Once suffering from APE, the patient's body will produce a variety of inflammatory factors, thereby destroying the endothelium of the pulmonary vessels, resulting in the production and activation of platelets, thereby increasing the level of MPV [14]. Gunay's team [15] conducted a study on 63 APE patients; their study found that compared with healthy people, the MPV level of APE patients was significantly increased, and MPV could effectively determine the disease situation of APE patients. Araz et al. [16] reported that among PE patients, the MPV level of dead patients was generally higher than that of survival patients, and the MPV level of relapsed patients was generally higher than that of nonrelapsed patients. The results showed that MPV has a certain role in the evaluation of death and recurrence of PE. Plasma NT-ProBNP is a commonly used clinical detection index; it has high sensitivity and stability and is not interfered with by drugs. Plasma NT-ProBNP plays a key role in the diagnosis and evaluation of coronary heart disease, respiratory failure, and other diseases [17, 18]. The plasma NT-ProBNP level in healthy people is low, and because the cardiomyocytes of APE patients are damaged, the pulmonary circulatory resistance increases, and the secretion of humoral factors increases, causing lung contraction, resulting in increased ventricular wall tension, thereby producing more NT-ProBNP [19, 20]. Its content can reflect the area of embolized blood vessels and heart function and has a positive effect on the prognosis of APE patients [21]. The simplified Geneva scale is a scoring method for judging the risk of thrombosis. The scoring includes items such as advanced age, medical history, fracture, heart rate, and so on [22]. It is objective, comprehensive, and repeatable and does not require excessive reliance on objective examinations, which helps evaluate the prognosis of APE patients [23]. The application of the simplified Geneva scale in the diagnosis and treatment of APE has the following clinical significance. ① It can simplify and optimize the prognosis assessment procedure of acute pulmonary embolism, save the medical cost, and reduce the possible adverse reactions caused by examination. ② In primary hospitals, due to the limitation of patients' medical expenses and the incomplete popularization of large-scale medical equipment such as CT, the treatment and prognosis assessment of APE are more difficult. The application of a simplified Geneva scale will bring convenience to primary hospitals and benefit primary patients. In this study, MPV, plasma NT-ProBNP, and simplified Geneva scale in the poor prognosis group were higher than those in the good prognosis group. MPV, plasma NT-ProBNP, and simplified Geneva scale were all independent risk factors for the poor prognosis of APE patients. The results showed that MPV, plasma NT-ProBNP, and simplified Geneva scale are all related to the prognosis of APE patients.

In addition, the ROC curve results showed that the AUC of MPV, plasma NT-ProBNP, and simplified Geneva scale in predicting the prognosis of APE patients were 0.818 (95% CI 0.712–0.925), 0.762 (95% CI 0.634–0.891), and 0.749 (95% CI 0.618–0.879), respectively, and the AUC of MPV and plasma NT-ProBNP combined with simplified Geneva scale in predicting the prognosis of APE patients was 0.907 (95% CI 0.826–0.988). The results suggested that MPV, plasma NT-ProBNP, and simplified Geneva scale have a certain predictive value for the prognosis of APE. Compared with a single index, the combination of the three indexes has a significant improvement in predicting the prognosis of APE, which has better clinical value.

## 5. Conclusion

In summary, MPV, plasma NT-ProBNP, and simplified Geneva scale have a certain predictive value for the prognosis of APE. Compared with a single index, the combination of the three indexes has a significant improvement in predicting the prognosis of APE and has better clinical value. This study has the limitation of the small number of included cases, and the other influencing factors of patients were not comprehensively observed. Therefore, we need to collect a larger sample of cases for further verification in the future and exclude other factors for a comprehensive discussion of the prognosis.

## Figures and Tables

**Figure 1:** Comparison of clinical indexes between the two groups. Note: compared with the good prognosis group, ^*∗*^*P* < 0.05.

**Figure 2:** Comparison of clinical scores between the two groups. Note: compared with the good prognosis group, ^*∗*^*P* < 0.05.

**Figure 3:** Prognostic value of each index in patients with APE.

**Table 1:** Simplified Geneva scale score.

Indexes	Score
Age ≥65 years old	1 point
Previous history of venous thrombosis or PE	1 point
History of surgery or lower limb fracture in the past 1 month	1 point
Active malignant tumor (entity or blood, currently active or cured within 1 year)	1 point
Unilateral lower limb pain	1 point
Hemoptysis	1 point
Heart rate, 75–94 beats/min	1 point
Heart rate, ≥95 beats/min	2 points
Unilateral deep vein tenderness and edema of the lower extremity	1 point

**Table 2:** Comparison of clinical data between the two groups (*n*, %, $\bar{x}\pm s$).

Clinical data	Good prognosis group (*n* = 45)	Poor prognosis group (*n* = 23)	*χ* ^2^/*t* value	*P* value
Age (years)	55.48 ± 11.26	57.71 ± 12.33	0.748	0.457
Gender				
Males	25 (55.56%)	14 (60.87%)	0.176	0.675
Females	20 (44.44%)	9 (39.13%)		
BMI (kg/m^2^)	23.90 ± 3.64	24.25 ± 3.87	0.367	0.714
Smoking history				
Yes	23 (51.11%)	13 (56.52%)	0.179	0.672
No	22 (48.89%)	10 (43.48%)		
Drinking history				
Yes	24 (53.33%)	15 (65.22%)	0.879	0.349
No	21 (46.67%)	8 (34.78%)		
Predisposing factors				
Deep vein thrombosis	14 (31.11%)	13 (56.52%)	4.105	0.043
Surgery or trauma	11 (24.44%)	2 (8.70%)	2.441	0.118
Tumor	4 (8.89%)	1 (4.35%)	0.461	0.497
Idiopathic	16 (35.56%)	7 (30.43%)	0.178	0.672
Primary diseases				
Diabetes	3 (6.67%)	6 (26.09%)	4.998	0.025
Hypertension	10 (22.22%)	3 (13.04%)	0.829	0.362
Hyperlipidemia	2 (4.44%)	5 (21.74%)	4.930	0.026
Coronary heart disease	9 (20.00%)	4 (17.39%)	0.067	0.797
Chronic kidney disease	7 (15.56%)	2 (8.70%)	0.624	0.429
Other diseases	14 (31.11%)	3 (13.04%)	2.649	0.103

**Table 3:** Multivariate analysis of prognostic factors in patients with APE.

Variable	*B* value	SE value	Wald value	OR value	95% CI	*P* value
PLT	1.068	0.577	3.426	2.909	0.939–9.015	0.078
PDW	1.374	0.428	10.306	3.951	1.708–9.142	0.017
MPV	1.907	0.462	17.038	6.732	2.722–16.651	0.004
Plasma NT-ProBNP	1.483	0.506	8.589	4.406	1.634–11.878	0.039
Simplified Geneva scale	1.820	0.653	7.768	6.172	1.716–2.495	0.042

**Table 4:** Prognostic value of each index in patients with APE.

Indexes	AUC	SE value	Asymptotically 95% CI		Optimal cutoff value	Sensitivity (%)	Specificity (%)
			Lower limit	Upper limit			
MPV	0.818	0.054	0.712	0.925	0.571	77.1	80.0
Plasma NT-ProBNP	0.762	0.065	0.634	0.891	0.475	71.5	76.0
Simplified Geneva scale	0.749	0.067	0.618	0.879	0.469	82.9	64.0
MPV + plasma NT-ProBNP + simplifiedGeneva scale	0.907	0.041	0.826	0.988	0.726	88.6	84.0

## Data Availability

The data used to support the findings of this study are available from the corresponding author upon request.
